The article "Endoplasmic reticulum stress promotes autophagy and apoptosis and reverses chemoresistance in human ovarian cancer cells" was retracted in 2025. Reasons: plagiarized images; duplicated images; overlap with other authors' work.

# Endoplasmic reticulum stress promotes autophagy and apoptosis and reverses chemoresistance in human ovarian cancer cells

**DOI:** 10.18632/oncotarget.17673

**Published:** 2017-05-07

**Authors:** Jin-Long Hu, Xin-Long Hu, Ai-Ye Guo, Chao-Jie Wang, Yi-Yang Wen, Shun-Dong Cang

**Affiliations:** ^1^ Department of Oncology, Henan Provincial People's Hospital, Zhengzhou 450000, P. R. China; ^2^ Department of Medical Imaging Technology, Henan University of Chinese Medicine, Zhengzhou 450000, P. R. China; ^3^ Laboratory of Clinical Research, Henan Provincial People's Hospital, Zhengzhou 450000, P. R. China

**Keywords:** endoplasmic reticulum stress (ERS), ovarian cancer, PI3K/AKT/mTOR, autophagy, apoptosis

## Abstract

Ovarian cancer presents the highest mortality rate among gynecological tumors. Here, we measured cell viability, proliferation, apoptosis, autophagy, and expression of endoplasmic reticulum stress (ERS)-related proteins, PI3K/AKT/mTOR pathway-related proteins, and apoptosis- and autophagy-related proteins in SKOV3 and SKOV3/CDDP cells treated with combinations of CDDP, tunicamycin, and BEZ235 (blank control, CDDP, CDDP + tunicamycin, CDDP + BEZ235, and CDDP + tunicamycin + BEZ235). Increasing concentrations of tunicamycin and CDDP activated ERS in SKOV3 cells, reduced cell viability and proliferation, increased apoptosis and autophagy, enhanced expression of ERS-related proteins, and inhibited expression of PI3K/AKT/mTOR pathway-related proteins. CDDP, tunicamycin, and BEZ235 acted synergistically to enhance these effects. We also detected lower expression of the ERS-related proteins caspase-3, LC3 II and Beclin 1 in ovarian cancer tissues than adjacent normal tissues. By contrast, expression of Bcl-2 and PI3K/AKT/mTOR pathway-related proteins was higher in ovarian cancer tissues than adjacent normal tissues. Lastly, expression of the ERS-related proteins Beclin 1, caspase-3 and LC3 II was higher in the sensitive group than the resistant group, while expression of Bcl-2, LC3 I, P62 and PI3K/AKT/mTOR pathway-related proteins was decreased. These results show that ERS promotes cell autophagy and apoptosis while reversing chemoresistance in ovarian cancer cells by inhibiting activation of the PI3K/AKT/mTOR signaling pathway.

## INTRODUCTION

Ovarian cancer is one of the most common cancers in women and is the leading cause of death from gynecologic malignancies [1]. Due to the subtlety of symptoms in its early stages, ∼75% of women are diagnosed with advanced disease at initial diagnosis [1]. For advanced ovarian cancer, the currently recommended management is primary cytoreductive surgery followed by platinum-paclitaxel combination chemotherapy [2]. The large failure rate of chemotherapy in treating patients with advanced disease contributes to poor prognosis [3].

The endoplasmic reticulum (ER) is a system of cisternae in the cytoplasm of many cells. Cell apoptosis and autophagy trigger the unfolded protein response, which can result in physiological or molecular disturbances that activate ER Stress (ERS) [4, 5]. ERS occurs in a variety of tumors and correlates with tumor cell survival and resistance to treatment [6]. ERS can activate autophagy while autophagy inhibition can enhance ERS-induced cell death [7]. Since ERS enhances tumor cell apoptosis, ERS activation could be exploited for therapeutic benefit against cancer [8].

The PI3K/AKT/mTOR signaling pathway is a classic pathway that promotes angiogenesis and cell progression [9, 10]. The PI3K/Akt/mTOR pathway has also been implicated in the development of several tumors [11, 12]. Inhibition of the PI3K/Akt/mTOR pathway has been reported to promote autophagy and apoptosis [13]. In most malignant tumors, this pathway is constitutively active, thereby promoting cell survival [14]. BEZ235 is a dual PI3K/mTOR inhibitor that can reverse resistance to CDDP [15]. Tunicamycin acts as an antibiotic that suppresses the intracellular production of N-linked glycans and can be used to induce ERS [16, 17]. Although previous studies have suggested that ERS was highly induced in various tumors and correlated with cancer cell survival and resistance to anti-cancer treatments [18, 19], few studies have explored the effect of ERS on human ovarian cancer cells. In this study, we used the ovarian cancer cell line SKOV3 and the drug-resistant cell lines SKOV3/CDDP to explore the relation of ERS and the PI3K/AKT/mTOR signaling pathway with autophagy, apoptosis and chemoresistance of SKOV3 and SKOV3/CDDP.

## RESULTS

### Tunicamycin induced the ERS in SKOV3 cells

We used tunicamycin to induce ERS in this study, as commonly done in other previous studies. Figure 1A shows cell viability of different cell lines using 1 mg/L tunicamycin for 24 h. The viability of SKOV3 cells was higher than that of SW626, HO8910, A2780 and 3AO cells (all *P* < 0.05). Therefore, we used SKOV3 cells in subsequent experiments. We used different concentrations of tunicamycin (0, 0.5, 1, 1.5 mg/L) to induce ERS in SKOV3 cells and measured its effect on growth after 12, 24, 48 and 72 h, using MTT assay. We found that tunicamycin inhibited the growth of SKOV3 cells in a concentration-dependent manner (Figure 1B). Cell vitality reached 50% at 1 mg/L tunicamycin for 24 h. Thus, we used such concentration and incubation time in experiments testing for the effects of CDDP and BEZ235 on ERS, the PI3K/AKT/mTOR signaling pathway, autophagy, proliferation and apoptosis.

**Figure 1:** Effects of tunicamycin on the viability of human ovarian cancer cells determined by MTT assay (**A**) Cell viability of different cell lines using 1 mg/L tunicamycin after 24 h; *P < 0.05 compared with the SKOV3 cells. (**B**) SKOV3 cell viability using different concentrations of tunicamycin (0, 0.5, 1, 1.5 mg/L); Tun, tunicamycin; *P < 0.05 compared with the 0 mg/L group at the same time; ^Δ^*P* < 0.05 compared with the same concentration group after 12 h. ^^^*P* < 0.05 compared with the same concentration group after 24 h; ^#^*P* < 0.05 compared with the same concentration group after 48 h. The experiments were performed three times and the average values were obtained.

### Tunicamycin induced ERS and inhibited the PI3K/AKT/mTOR signaling pathway in a concentration-dependent manner in SKOV3 cells

Figure 2A shows the expression of ERS-related proteins CHOP, PERK, PDI and Grp78 in SKOV3 cells treated with different concentrations of tunicamycin (0, 0.5, 1, 1.5 mg/L). The expression of these proteins increased gradually with increasing concentrations of tunicamycin. Conversely, the expression of PI3K, AKT, mTOR, p-PI3K, p-AKT and p-mTOR decreased, indicating that tunicamycin treatment induced ERS in SKOV3 cells and inhibited the PI3K/AKT/mTOR pathway (Figure 2B).

**Figure 2:** Expressions of ERS-related proteins and PI3K/AKT/mTOR pathway-related proteins after SKOV3 cells were treated by different concentrations of tunicamycin (0, 0.5, 1, 1.5 mg/L) for 24 h (**A**) Expressions of CHOP, PERK, PDI and Grp78 proteins. (**B**) the expressions of PI3K, AKT, mTOR, p-PI3K, p-AKT and p-mTOR. *P < 0.05 compared with the 0 mg/L group; the experiments were performed three times and the average values were obtained.

### Tunicamycin inhibited proliferation while promoting autophagy and apoptosis in SKOV3 cells

In order to further study autophagy and apoptosis in SKOV3 cells treated with different concentrations of tunicamycin (0, 0.5, 1, 1.5 mg/L) for 24 h, we measured the expression of autophagy-related proteins (LC3 I, LC3 II, P62 and Beclin 1) and apoptosis-related proteins (procaspase-3, caspase-3 and Bcl-2) in each group (Figure 3A). The expression of Beclin 1 and caspase-3 increased with increasing tunicamycin concentration while the expression of P62 and Bcl-2 decreased gradually. Furthermore, LC3 I was converted to LC3 II and procaspase-3 was activated. Hochst33342/PI staining showed that with increasing tunicamycin concentration, the number of apoptotic cells increased gradually while the ratio of necrotic cells remained the same (Figure 3B). Annexin V-FITC/PI staining also showed increased apoptosis rates with increasing tunicamycin concentration (Figure 3C). Colony formation assay indicated that increasing concentrations of tunicamycin reduced SKOV3 proliferation (Figure 3D). MDC staining showed that increasing concentrations of tunicamycin gradually increased autophagy (Figure 3E). Taken together, these results demonstrated that tunicamycin treatment induced autophagy and apoptosis in SKOV3 cells.

**Figure 3:** Comparisons of the autophagy, proliferation and apoptosis after SKOV3 cells were treated by different concentrations of tunicamycin (0, 0.5, 1, 1.5 mg/L) for 24 h (**A**) Expressions of apoptosis-related proteins (procaspase-3, caspase-3 and Bcl-2) and autophagy-related proteins (LC3 I, LC3 II, P62 and Beclin 1). (**B**) Percentage of apoptotic cells and necrotic cells measured by Hochst33342/PI staining. (**C**) Apoptosis rate measured by annexin V-FITC/PI staining. (**D**) Proliferation measured by colony formation assay. (**E**) Autophagy measured by MDC staining. *P < 0.05 compared with the 0 mg/L group. The experiments were performed three times and the average values were obtained.

### Tunicamycin increased the sensitivity of SKOV3 cells to CDDP

SKOV3 cells in the logarithmic growth phase were treated with increasing concentrations of CDDP (0, 0.5, 1, 1.5 μg/mL). After 12, 24, 48 and 72 h, cell viability was measured by MTT assay to quantify the sensitivity of SKOV3 cells to CDDP. We found that CDDP decreased cell viability. However, CDDP resistance developed with increasing incubation time, reducing the sensitivity of SKOV3 cells to CDDP over time (Figure 4A). Cells in the logarithmic growth phase were supplemented with 1 mg/L tunicamycin and with different concentrations of CDDP (0, 0.5, 1, 1.5 μg/mL) after 24 h. We measured cell viability using MTT assay 12, 24, 48 and 72 h after addition of CDDP to quantify CDDP resistance in SKOV3 cells under ERS. Cell viability decreased after CDDP was added in each group in a concentration- and time-dependent manner (Figure 4B). When IC50 was 1.199 ± 0.079 μg/mL, SKOV3 cells showed the greatest sensitivity (and the least resistance) to chemotherapeutic CDDP after tunicamycin-induced ERS.

**Figure 4:** Cell viability under different concentrations of CDDP (0, 0.5, 1, 1.5 μg/mL) without tunicamycin treatment and after SKOV3 cells were treated by tunicamycin for 24 hours Note: (**A**) Cell viability of SKOV3 cells treated by CDDP (0, 0.5, 1, 1.5 μg/mL); (**B**) cell viability of SKOV3 cells treated by CDDP (0, 0.5, 1, 1.5 μg/mL) after 24 hours of tunicamycin; *P < 0.05 compared with the 0 μg/mL CDDP group at the same time or the result at 12 h with the same concentration; ^Δ^*P* < 0.05 compared with the 0.5 μg/mL CDDP group at the same time or the result at 24 h with the same concentration; ^^^*P* < 0.05 compared with the 1 μg/mL CDDP group at the same time or the result at 48 h with the same concentration; ^#^*P* < 0.05 compared with the 1.5 μg/mL CDDP group at the same time or the result at 72 h with the same concentration; the experiments were performed three times and the average values were obtained.

### Tunicamycin combined with CDDP induced ERS and inhibited the PI3K/AKT/mTOR signaling pathway in SKOV3 cells

SKOV3 cells in each group were supplemented with 1 mg/L tunicamycin and incubated for 24 h. Then, the cells were treated with increasing concentrations of CDDP (0, 0.5, 1, 1.5 μg/mL) and incubated for another 24 h. The expression of ERS-related proteins CHOP, PERK, PDI and Grp78 in each group increased with increasing concentrations of CDDP (Figure 5A). On the other hand, the expression of PI3K, AKT, mTOR, p-AKT and p-mTOR in each group decreased gradually with increasing concentrations of CDDP (Figure 5B). These results indicated that CDDP promoted ERS and inhibited the PI3K/AKT/mTOR pathway in SKOV3 under tunicamycin-induced ERS.

**Figure 5:** Expressions of ERS-related proteins and PI3K/AKT/mTOR pathway-related proteins under different concentrations of CDDP (0, 0.5, 1, 1.5 μg/mL) after SKOV3 cells were treated by 1 mg/L tunicamycin (**A**) Expression of ERS-related proteins CHOP, PERK, PDI and Grp78. (**B**) Expression of PI3K, AKT, mTOR, p-PI3K, p-AKT and p-mTOR. *P < 0.05 compared with the 0 mg/L group. The experiments were performed three times and the average values were obtained.

### Tunicamycin combined with CDDP inhibited proliferation while promoting autophagy and apoptosis in SKOV3 cells

The expression of caspase-3 and Beclin 1 in SKOV3 cells in each group increased after tunicamycin treatment (1 mg/L) and incubation (24 h). On the other hand, with increasing concentrations of CDDP, the expression of Bcl-2 and P62 decreased gradually, procaspase-3 was activated, and LC3 I was converted to LC3 II (Figure 6A). The apoptosis rate in each group gradually increased while the ratio of necrotic cells remained unchanged (Figure 6B–6C). Colony formation assay suggested that increasing concentrations of CDDP reduced the proliferation of SKOV3 cells (Figure 6D). MDC staining showed that after tunicamycin treatment, the autophagy rate increased gradually with increasing concentrations of CDDP (Figure 6E). This suggests that CDDP contributed to autophagy and apoptosis in SKOV3 cells.

**Figure 6:** The autophagy, proliferation and apoptosis of SKOV3 cells under different concentrations of CDDP (0, 0.5, 1, 1.5 μg/mL) after SKOV3 cells were treated by 1 mg/L tunicamycin for 24 h (**A**) Expressions of apoptosis-related proteins (procaspase-3, caspase-3 and Bcl-2) and autophagy-related proteins (LC3 I, LC3 II, P62 and Beclin 1). (**B**) Percentage of apoptotic cells and necrotic cells measured by Hochst33342/PI staining. (**C**) Apoptosis rate measured by annexin V-FITC/PI staining. (**D**) Proliferation measured by colony formation assay. (**E**) Autophagy measured by MDC staining. *P < 0.05 compared with the 0 mg/L group. The experiments were performed three times and the average values were obtained.

### BEZ235 activated ERS and inhibited the PI3K/AKT/mTOR pathway in SKOV3/CDDP cells

We treated CDDP-resistant cells SKOV3/CDDP with the PI3K/AKT/mTOR pathway inhibitor BEZ235 and measured the expression of various ERS-related proteins, PI3K/AKT/mTOR pathway-related proteins, and p-PI3K, p-AKT and p-mTOR. In the presence of both tunicamycin and BEZ235, the expression of CHOP, PERK, PDI and Grp78 was higher than that in the CDDP + BEZ235 and the CDDP + tunicamycin groups (Figure 7A). On the other hand, the expression of PI3K/AKT/mTOR pathway-related proteins was lower in the CDDP + tunicamycin + BEZ235 group compared to that in other groups (Figure 7B). Taken together, these results suggested that inhibition of the PI3K/AKT/mTOR pathway could activate ERS.

**Figure 7:** Expressions of ERS-related proteins and PI3K/AKT/mTOR pathway-related proteins in SKOV3/CDDP cells among five groups (**A**) Expression of ERS-related proteins CHOP, PERK, PDI and Grp78. (**B**) Expression of PI3K, AKT, mTOR, p-PI3K, p-AKT and p-mTOR. *P < 0.05 compared with the blank control group; ^#^*P* < 0.05 compared with the CDDP+tunicamycin group; ^Δ^*P* < 0.05 compared with the CDDP+ BEZ235 group. The experiments were performed three times and the average values were obtained.

### BEZ235 inhibited proliferation while promoting autophagy and apoptosis in SKOV3/CDDP cells

We measured autophagy and apoptosis in SKOV3/CDDP cells and control cells under various treatments. CDDP + tunicamycin treatment activated apoptosis-related protein pro-caspase-3 while increasing the expression of caspase-3 and decreasing the expression of Bcl-2. These effects were enhanced by addition of BEZ235 (Figure 8A). CDDP + tunicamycin treatment also increased the expression of autophagy-related protein Beclin 1, decreased the expression of P62, and resulted in the conversion of LC3 I to LC3 II. These effects were enhanced by BEZ235 (Figure 8B). Proliferation decreased in cells treated with CDDP + tunicamycin + BEZ235 compared to controls, but was higher than that in cells created with CDDP + tunicamycin or CDDP + BEZ235. Furthermore, annexin V-FITC/PI staining showed a higher percentage of apoptotic cells in the CDDP + tunicamycin + BEZ235 group compared to controls and to the CDDP + tunicamycin and CDDP + BEZ235 groups (Figure 8C, 8D). MDC staining showed that autophagy was also higher in the CDDP + tunicamycin + BEZ235 group than in other groups (Figure 8E). These results demonstrated that inhibition of the PI3K/AKT/mTOR pathway induced autophagy and apoptosis in SKOV3/CDDP cells.

**Figure 8:** Comparisons of autophagy, proliferation and apoptosis of SKOV3/CDDP cells in five groups (**A**) Expression of apoptosis-related proteins (procaspase-3, caspase-3 and Bcl-2) and autophagy-related proteins (LC3 I, LC3 II, P62 and Beclin 1). (**B**) Percentage of apoptotic cells and necrotic cells detected by Hochst33342/PI staining. (**C**) Apoptosis rate measured by annexin V-FITC/PI staining. (**D**) Proliferation measured by colony formation assay. (**E**) Autophagy measured by MDC staining. *P < 0.05 compared with the blank control group; ^#^*P* < 0.05 compared with the CDDP group; ^Δ^*P* < 0.05 compared with the CDDP + tunicamycin group. The experiments were performed three times and the average values were obtained.

### Ovarian cancer tissues sensitive to chemotherapy showed ERS, increased autophagy and apoptosis, and inhibition of the PI3K/AKT/mTOR pathway

Western blotting indicated that, compared to adjacent normal tissues, the expression of CHOP, PERK, PDI, Grp78, caspase-3, and P62 was increased in ovarian cancer tissues. On the other hand, expression of PI3K, AKT, mTOR, Bcl-2, and Beclin 1 was decreased (all *P* < 0.05) (Figure 9). Compared to the resistant group, the expression of CHOP, PERK, PDI, Grp78, caspase-3, and Beclin 1 was increased in the sensitive group. On the other hand, the expression of PI3K, AKT, mTOR, p-PI3K, p-AKT, p-mTOR, P62, and Bcl-2 was decreased. Furthermore, procaspase-3 was activated, the expression of autophagy-related protein decreased, and LC3 I was converted to LC3 II (all *P* < 0.05) (Figure 10).

**Figure 9:** Expression of ERS-related proteins, PI3K/AKT/mTOR pathway-related proteins, autophagy-related proteins, and apoptosis-related proteins in ovarian cancer tissues and adjacent normal tissues *P < 0.05 compared with the ovarian cancer tissues. The experiments were performed three times and the average values were obtained.

**Figure 10:** Expression of ERS-related proteins, PI3K/AKT/mTOR pathway-related proteins, autophagy-related proteins and apoptosis-related proteins in the resistance group and sensitive group (**A**) Expression of ERS-related proteins CHOP, PERK, PDI and Grp78 in the resistance group and sensitive group. (**B**) Expression of PI3K, AKT, mTOR, p-PI3K, p-AKT and p-mTOR in the resistance group and sensitive group. Expressions of apoptosis-related proteins (procaspase-3, caspase-3 and Bcl-2) and autophagy-related proteins (LC3 I, LC3 II, P62 and Beclin 1). *P < 0.05 compared with the resistance group. The experiments were performed three times and the average values were obtained.

## DISCUSSION

Ovarian cancer has the highest mortality among gynecological tumors [1]. CDDP administration is the first line of treatment for ovarian cancer, but resistance and adverse side effects limit its clinical application [20]. Muilenburg *et al*. found that autophagy and apoptosis inhibit development and reduce drug resistance in pancreatic cancer, thereby improving prognosis [21]. Therefore, understanding the mechanism of signaling pathways related to ovarian cancer can help to minimize drug resistance and improve clinical treatment.

In this study, we found that the tunicamycin could activate ERS and inhibit the PI3K/AKT/mTOR signaling pathway in SKOV3 cells, thereby enhancing apoptosis and autophagy. Tunicamycin is an antibiotic that can kill bacteria, fungi and viruses by inhibiting the glucosylation of proteins and inducing ERS [22]. Under ERS, cells present endoplasmic reticulum with unfolded or wrongly folded proteins, which promotes the expression of protein disulfide isomerase (PDI) [23]. Here, we also found that increasing concentrations of tunicamycin increased the expression of PDI and Grp78 while activating ERS. Grp78 is known to induce ERS [24]. ERS induces cell apoptosis by activating transcription factors CHOP/GADD153, the kinase pathway ASK1/JNK, and Caspase-2 [25]. ERS also promotes autophagy by inducing Ca^2+^ release from the endoplasmic reticulum into the cytoplasm and activating various kinases and proteases [26]. Tunicamycin inhibits N-glycosylation and causes ERS and toxicity in normal tissues [27]. The activation of PERK and CHOP result in the upregulation of ER protein folding capacity and ER-associated degradation [28]. CHOP is one of the downstream components in the unfolded protein response (UPR)-mediated apoptotic pathway in response to ERS [29]. CHOP also activates caspase-3 [30]. The PI3K/AKT/mTOR is a signaling pathway that promotes cell proliferation, metabolism and survival, and is commonly deregulated in various types of cancer [31]. Alterations of the PI3K/AKT/mTOR signaling pathway lead to PI3K activation and malignant transformation [32]. mTOR is a serine/threonine protein kinase that promotes cell growth, motility and survival, and dysregulation of the mTOR signaling pathway is observed in many types of cancer [33]. Previous study has shown that ERS can negatively regulate the AKT/TSC/mTOR signaling pathway to promote autophagy [34], in agreement with the results of our present study.

Inhibition of the PI3K/AKT/mTOR signaling pathways induces cell apoptosis, increases the expression of caspase-3, and decreases the expression of Bcl-2. The PI3K/AKT/mTOR signaling pathway is activated in many different cancers [12]. Beclin 1 is essential for autophagy induction and other biological processes [35]. LC3 is present in autophagosomes, and serves as a widely used marker for autophagosomes [36]. Mammalian target of rapamycin (mTOR) is a master regulator of cell growth versus autophagy [37]. For these reasons, inhibition of the PI3K/AKT/mTOR signaling pathways induces autophagy, and enhances the expressions of Beclin1 and LC3. Caspase-3 initiates apoptosis [38]. When caspase-3 increases, the PI3K/AKT pathway is activated and inhibits apoptosis [39].

Our experiments here showed that the PI3K/AKT/mTOR pathway was inhibited while apoptosis and autophagy were promoted after adding CDDP to SKOV3 cells treated with tunicamycin. Akt is a serine/threonine kinase that promotes tumor cell growth by phosphorylating transcription factors such as YB-1 and cell cycle proteins [40]. Previous studies also showed that the PI3K/AKT/mTOR pathway reduced the sensitivity of tumor cells to chemotherapy [41, 42]. CDDP is a frequently used chemotherapeutic drug that can cause ototoxicity and nephrotoxicity at high doses [43]. CDDP can cross-link to DNA, thereby inhibiting replication and transcription [44]. Once DNA is damaged, cell cycle check points are activated, delaying cell cycle progression, which triggers either DNA repair or apoptosis [45] Yu XS *et al*. demonstrated that CDDP could induce ERS and apoptosis [46]. AKT regulates multiple downstream targets, resulting in cell growth, survival and CDDP resistance [47]. CDDP was reported to activate the PI3K/AKT signaling and lead to CDDP resistance in ovarian cancer [48]. Qin L *et al*. demonstrated that CDDP could induce protective autophagy, which resulted in decreased sensitivity to chemotherapy [49].

The PI3K/AKT/mTOR pathway inhibitor BEZ235 promotes ERS, inducing cell autophagy and apoptosis in many cancer cell lines [50, 51]. PS Yeh *et al*. found that the PI3K/AKT pathway inhibited apoptosis as a result of resistance to ERS [52]. The aforementioned studies are consistent with the results of our present study, showing that the expression of autophagy-related proteins LC3 and Beclin 1 and of apoptosis-related proteins caspase-3 is increased in the presence of BEZ235 while the expression of apoptosis-suppressing protein Bcl-2 is inhibited. BEZ235 eliminates the feedback activation of PI3K activity due to mTOR inhibition and is therefore a promising therapeutic target [53]. Indeed, a previous study found that BEZ235 inhibited tumor proliferation by downregulating the PI3K/AKT/mTOR signaling pathway [54].

Our study suffers from some limitations. First, whether tunicamycin treatment alone increases MDC staining needs to be further verified. Second, the effects of autophagy on ovarian cancer cells should be further characterized. Nonetheless, the results of our experiments indicate that ERS promotes autophagy and apoptosis and reverses chemoresistance of ovarian cancer SKOV3 cells via inhibition of the PI3K/AKT/mTOR signaling pathway.

## MATERIALS AND METHODS

### Study subjects

Between August 2012 and June 2015, 108 ovarian cancer patients between 21 and 75 years old (median 51) were recruited from the People's Hospital of Zhengzhou University and Henan Provincial People's Hospital to participate in our study. We obtained ovarian cancer tissues and adjacent normal tissues from each patient. All the patients received comprehensive staging surgery at the early stage or satisfactory cytoreductive surgery and platinum-based chemotherapy after surgery. Follow-ups were conducted among patients that met requirements, including the sensitive group with 65 patients (platinum-based chemotherapy reached clinical remission with recurrence after stopping chemotherapy for over six months) and the resistance group with 43 patients (with recurrence in six months after stopping chemotherapy). Inclusion criteria: patients received the first treatment in our hospital; patients received comprehensive staging surgery at the early stage or satisfactory cytoreductive surgery; ovarian cancer was verified by postoperative pathology; patients received platinum-based chemotherapy after surgery; follow-up data were complete. Exclusion criteria: patients had a history of other malignant tumors; patients without comprehensive staging surgery or satisfactory cytoreductive surgery; patients received adjuvant therapy such as radiotherapy and chemotherapy before surgery; metastatic ovarian tumors were eliminated; follow-up data were incomplete. This study was approved by the Ethical Committee of the People's Hospital of Zhengzhou University and Henan Provincial People's Hospital. Written informed consent was acquired from all study subjects at the time of hospitalization to undergo diagnostic and therapeutic procedures. This study complied with the guidelines and principles of the Declaration of Helsinki [55].

### Cell culture and grouping

Human ovarian cancer SKOV3, SW626, HO8910, A2780 and 3AO cell lines and CDDP-resistant SKOV3/CDDP cell lines were taken from the cell bank of the People's Hospital of Zhengzhou University and Henan Provincial People's Hospital and cultured by RPMI-1640 medium containing 10% fetal bovine serum (FBS). Cells were cultured in an incubator (Sanyo, Japan) at 37°C, 5% CO_2_ and 90% relative humidity. Then, the cells were digested with 0.4% trypsin for passage. CDDP (1 μg/mL) was added in the medium of SKOV3/CDDP cell lines to maintain the chemoresistance of cells. SKOV3/CDDP cells were divided into the following four groups: (1) CDDP group (only treated with CDDP); (2) CDDP + tunicamycin group (treated with 1 mg/L tunicamycin, then with CDDP); (3) CDDP + BEZ235 (Selleck Chemicals, the United States) group (treated with CDDP, then with 5 μmol/L BEZ235); (4) CDDP + BEZ235 + tunicamycin group (treated with 1 mg/L tunicamycin, then with CDDP and 5 μmol/L BEZ235). Each index was measured at the 24th hour after drugs were added in each group. SKOV3 cells were used as the blank control group.

### MTT assay for cell viability

SKOV3, SW626, HO8910, A2780 and 3AO cells in the logarithmic growth phase were collected and seeded in a 96-well plate at a density of 8 × 10^4^ cells per well. Adherent cells were supplemented with 1 mg/L tunicamycin and cultured for 24 h. We added 20 uL MTT (Sigma, USA) (5 mg/L) into each well and cultured the cells further for 4 h. The liquid was sucked out and 150 uL dimethylsulfoxide were added, shaking for 10 min. An enzyme-labeled instrument (Beckman, the United States) was used to measure the optical density of cells at 490 nm and 570 nm.

Tunicamycin (0, 0.5, 1 and 1.5 mg/L) was added into SKOV3 cells separately, followed by incubation for another 24 h. After 20 uL MTT (Sigma, USA) (5 mg/mL) was added into each well, the cells were cultured for an additional 4 h. The liquid was extracted, 150 uL dimethylsulfoxide were added, and the culture was shaken for 10 min. The optical density of the cells in each group was measured at 490 nm and 570 nm using an enzyme-labeled instrument (Beckman, the United States). Cells in the CDDP + tunicamycin group (1 mg/L) were supplemented with 0, 0.5, 1 and 1.5 μg/mL CDDP l to culture for 24 h before detecting.

### Colony formation assay

SKOV3 and SKOV3/CDDP cells in the logarithmic growth phase were digested with trypsin, centrifuged at 1000 r/min for 5 min and supplemented with serum-free medium for single cell suspension. After counting, 1000 cells were obtained from each group and separately added into a 6-well plate with medium at 37°C, turning the plate to make the cells separated. Cells were placed in an incubator with 5% CO_2_ and saturated humidity at 37°C for 2∼3 weeks of culture. The growth of cells was monitored and the medium was replaced timely. When there was visible colony formation in the culture dish, the culture was terminated. After removing the supernatant, the cells were washed twice with phosphate buffer saline (PBS) and fixed in 5 mL paraformaldehyde for 15 min. With removal of fixative solution, cells were washed with PBS twice, stained with Giemsa for 15 min, and then washed with running water to remove the staining solution with air-drying. The colony number was counted under a microscope (low power). More than 50 cells were considered as a clone.

### Hoechst3334/PI staining

The apoptosis rates of SKOV3 and SKOV3/CDDP cells were measured using Hoechst33342/PI kit (Sigma, USA). Cells in logarithmic growth phase were seeded onto a 24-well plate with 1 cm × 1 cm sterile glass slides at a density of 5 × 10^4^ cells per well, and cultured for another 24 h after the cells were adherent. On the next day, cells were rinsed three times using 0.1 mol/L PBS, and fixed in 4% paraformaldehyde for 25 min at room temperature. Then, the cells were rinsed three times again, and supplemented with a mixture containing 1 mL PBS, 1 mL Hoechst33342 and 100 mL PI at room temperature for 5 min. Then, the cells were rinsed three times, and sealed using a fluorescence-quenching agent in the dark. The cells were examined and imaged with a laser confocal microscope (Olympus, Japan). Apoptotic cells were light blue and necrotic cells were red under the microscope. To measure the percentage of apoptotic cells and necrotic cells, three fields were selected from each sample randomly. In each field, 500 cells were counted to calculate the percentage of average apoptotic cells and necrotic cells as apoptosis rate and necrosis rate.

### Annexin V-FITC/PI staining

After 48 h, cells were digested with trypsin without EDTA, collected in flow tubes and centrifuged at 1000 r/min for 5 min, with removal of the supernatant. Cells were washed with PBS 3 times and centrifuged to remove the supernatant. According to the instructions of Annexin V-FITC Apoptosis Detection kit (Sigma, USA), cells in each tube were supplemented with 150 μL binding buffer and 5 μL Annexin-V-FITC, shaken, mixed and cultured at room temperature for 15 min in the dark. Then, the cells were shaken and mixed with addition of 100 μL binding buffer and 5 μL PI (Sigma, USA). Flow cytometry was used to measure cell apoptosis. Cells in the left lower quadrant were normal cells while early apoptotic cells were in the right lower quadrant, late apoptotic cells in the right upper quadrant, and dead cells in the left upper quadrant.

### MDC staining

The SKOV3 and SKOV3/CDDP cells in each group were seed to a 6-well plate at a density of 1 × 10^6^ cells per well. Adherent cells were added with drugs and cultured for another 24 h. On the next day, after being digested and collected, the cells were rinsed twice with PBS after centrifugation. The supernatant was discarded. The cells were suspended in 300 μL PBS, supplemented with 3 μL MDC and cultured for 30 min at 37°C. After rinsing with PBS, the cells were centrifuged into sedimentation, supplemented with 1 mL 4% paraformaldehyde and incubated in dark place for 15 min. The cells were rinsed again, centrifuged and then supplemented with 500 μL buffer for resuspension. A fluorescence microscope (Olympus, Japan) was used to visualize the cells. From each sample, 1 × 10^4^ cells were collected. CellQuest software was used to collect data. The result was expressed as the percentage of autophagy.

### Western blotting

Using Bioford method, we measured protein concentration in SKOV3 and SKOV3/CDDP cells, as well as in ovarian cancer tissues and adjacent normal tissues for each group. We used SDS-PAGE and we calculated the sample size according to the protein concentration. The samples were blended with buffer at 1:1 and bathed in boiling water for 5 min. Then, 5% stacking gel and 12% separating gel were used for electrophoresis under 80 V and 100 V, respectively. The gel was cut and tagged at one angle. The “sandwich” was compounded and trans-membraned using 200 mA steady current for 2 h in a 4°C cold room. After being blocked with 5% skimmed milk powder for 1 h at room temperature, membranes were washed with TBST 3 times, each time for 10 min. Then, the samples were supplemented with the following primary antibodies: anti-CHOP, anti-PERK, anti-PDI, anti-Grp78, anti-PI3K, anti-p-PI3K, anti-AKT, anti-p-AKT, anti-mTOR, anti-p-mTOR, anti-procaspase-3, anti-Caspase-3, anti-Bcl-2, anti-LC3 I, anti-LC3 II, anti-Beclin1, anti-P62 and anti-β-actin (Abcam, the United States), and incubated overnight at 4°C. On the next day, the membranes were washed with TBST three times for 10 min each time. Then the samples were incubated with HRP-labeled goat anti-rabbit IgG (Sigma, USA) for 1 h at room temperature. After the membranes were washed, samples were stained by ECL kit (Beyotime Biotechnology, China) and scanned using a gel imaging system. ImageJ software was used to analyze the stripes. The relative expression of each target protein was measured using β-actin as an endogenous reference.

### Statistical analysis

SPSS 21.0 software (SPSS Inc., Chicago, IL, USA) was used for data analysis. The measurement data was expressed as mean ± standard deviation (SD). The two groups were compared using unpaired *t* test. Paired *t* test was used to compare different time points in the same concentration group. One-way analysis of variance (ANOVA) was used for multiple comparisons. *P* < 0.05 was considered statistically significant.
